# Study on the Antihypertensive Mechanism of* Astragalus membranaceus* and* Salvia miltiorrhiza* Based on Intestinal Flora-Host Metabolism

**DOI:** 10.1155/2019/5418796

**Published:** 2019-07-21

**Authors:** Cong Han, Yue-hua Jiang, Wei Li, Yao Liu, Zhen-qiang Qi

**Affiliations:** ^1^Shandong University of Traditional Chinese Medicine, Jinan 250014, China; ^2^Central Laboratory of Affiliated Hospital of Shandong University of Traditional Chinese Medicine, Jinan 250014, China; ^3^Nephropathy Department, Affiliated Hospital of Shandong University of Traditional Chinese Medicine, Jinan 250014, China

## Abstract

Our previous studies have shown that the combination of* Astragalus membranaceus* and* Salvia miltiorrhiza* (HD) had a good antihypertensive effect, but its potential mechanism remained unclear. This study aimed to investigate the role of intestinal flora and serum metabolism induced by HD against hypertension. 16 spontaneous hypertensive rats (SHRs) were divided into HD group (5.9 g/kg) and model group (M) (normal saline), with eight Wistar-Kyoto (WKY) rats as control group (W) (normal saline). Rats were fed by gavage once a day for 28 days. The changes of intestinal flora and serum metabolism were analyzed by 16S rDNA sequencing and LC-MS/MS assay. HD decreased blood pressure steadily, improved the structure and composition of imbalance flora in SHRs, increased the abundance and diversity of flora, and decreased flora Firmicutes to Bacteroidetes (F/B) ratio.* Rumen bacterium NK4A214, Clostridium *sp.* MC 40 *increased remarkably in M group.* Akkermansia, Akkermansia muciniphila, *and* Lactobacillus intestinalis *increased significantly in HD group, which were functionally related to the significant increase of* Lachnoclostridium*,* Faecalibaculum,* and* Lactobacillus reuteri* in W group, which were all probiotics producing butyric acid, lactic acid, and regulating inflammation and other antihypertensive related factors. HD also changed the serum metabolic pattern of SHRs. 16 potential biomarkers related to inflammation, vasodilation, steroid hormones, oxidative stress, and etc. changed significantly, mainly enriched in arachidonic acid metabolism, tryptophan metabolism, steroid hormone biosynthesis, and glutathione metabolism. The correlation analysis demonstrated that the dominant genius and species in three groups were highly correlated with steroid hormone biosynthesis, arachidonic acid metabolism, tryptophan metabolism, and vitamin B6 metabolism. Our research indicated that HD had a good antihypertensive effect, which may be driven by the protective intestinal flora and beneficial metabolites induced by it, and the metabolites were closely related to the changes of intestinal flora. It provided new insights for the antihypertensive mechanism of HD.

## 1. Introduction

The intestinal flora as the second genome of the human body was not only directly involved in the normal metabolism but also closely related to the occurrence and development of hypertension [1–6]. It had been found that both spontaneous hypertensive rats (SHRs) and hypertensive patients had the microecological imbalance of the richness, diversity, and uniformity in intestinal flora and the increased ratio of Firmicutes to Bacteroidetes [4]. In addition, a meta-analysis of multiple randomized human clinical trials had shown that probiotics could effectively lower blood pressure [5]. A recent study found that blood pressure was elevated by fecal transplantation from hypertensive human donors to germ-free mice. And their study also confirmed that serum metabolic changes in patients with prehypertension and hypertension were closely related to intestinal flora imbalance [6]. Metabolomics, as a powerful tool for identifying the changes of endogenous metabolites in pharmacodynamics, had been widely used in exploring the pathological mechanism of cardiovascular and cerebrovascular diseases such as hypertension in recent years [7]. The metabolic studies of SHRs had found that the changes of metabolites in the pathways of arachidonic acid metabolism, lipid metabolism, fatty acid metabolism, vitamin metabolism, and amino acid metabolism were closely related to the regulation of blood pressure [8–10]. However, the specific mechanism between intestinal flora-host metabolism and blood pressure regulation has not been fully elucidated.

*Astragalus membranaceus *(of the Leguminosae family), with Chinese name of Huang qi and the Latin name of* Astragalus membranaceus *(Fisch.) Bge., is well used in Traditional Chinese Medicines (TCM) for the treatment of general weakness to increase overall immunity.* Salvia miltiorrhiza *(of the Lamiaceae family), with Chinese name of Dan shen and the Latin name of* Salvia miltiorrhiza *Bge., is highly valued in TCM for activating blood circulation to dissipate blood stasis. Both of them have been widely used in the treatment of hypertension in China. It had been found that astragaloside IV, an effective component of* Astragalus membranaceus*, reduced blood pressure in rats with metabolic syndrome by regulating lipid metabolism and endothelium-dependent vasodilation [11].* Salvia miltiorrhiza* aqueous extract reduced blood pressure by inhibiting SHRs' vascular remodeling and oxidative stress [12]. The combination of* Astragalus membranaceus* and* Salvia miltiorrhiza *(HD) could reduce blood lipid and improve insulin resistance, anti-inflammation, and anticoagulation [13–15], all of which were risk factors of hypertension. Our previous studies had found that the combination of HD had better antihypertensive effect than the separated use of herb, but the pharmacological mechanism of blood pressure reduction remained to be further clarified.

Therefore, we speculate that the combination of HD may be involved in the regulation of blood pressure by inducing changes in intestinal flora and serum metabolites. In the present study, we performed 16S rDNA V4 region high throughput sequencing on intestinal flora and LC-MS/MS assay on serum metabolites and analyzed the correlation between intestinal flora and serum metabolism, to explore the potential antihypertensive mechanism of combination of HD.

## 2. Materials and Methods

### 2.1. Preparation of HD

HD were purchased from the Affiliated Hospital of Shandong University of Traditional Chinese Medicine (Jinan, China) and authenticated by Professor Chuanjiang Ma (Chief Pharmacist of Affiliated Hospital of Shandong University of Traditional Chinese Medicine). According to our previous studies and other reports [16], HD were prepared in a ratio of 2:1, adding 10-fold volume of water to the medicinal material, decocted twice, mixed, and concentrated to 0.59g of crude drug per ml.

### 2.2. Animal and Drug Administration

The research protocol was approved by the Animal Experimental Ethics Committee of the Affiliated Hospital of Shandong University of Traditional Chinese Medicine. Sixteen 16-week-old male SHRs were divided into two groups: HD group (HD) and model group (M) (n = 8) and eight male Wistar-Kyoto (WKY) rats of the same age as control group (W), all of which were purchased from Vital River Laboratory Animal Technology Co. Ltd. (Beijing, China) with animal license number SCXK (Beijing) 2016-0006. The HD group was intragastrically administrated with HD (0.59 g/mL, 10 mL/kg), and rats in M group and W group were administrated with the same amount of normal saline. All animals were fed by gavage once a day for 28 days.

### 2.3. Blood Pressure Measurement

The blood pressure of rats' tail artery was measured by noninvasive blood pressure meter before and 1, 2, 3, and 4 weeks after administration. The data were expressed by means ± SD, and multiple comparisons were performed by one-way analysis of variance (ANOVA) using SPSS 19.0 (SPSS Inc., USA).

### 2.4. Sample Collection and Preparation

*Serum Sample Preparation*. Rats were anesthetized by intraperitoneal injection of 3% pentobarbital sodium (40 mg/kg) and serum samples were collected from the abdominal aorta of each rat on the 28th day and immediately centrifuged at 3,000 rpm for 10 min. The supernatant was transferred into a clean tube and stored at −80°C. Prior to analysis, 100 uL serum was resuspended with prechilled 80% methanol (-20°C) followed by well vortexing. The samples were incubated at −20°C for 60 min and then were centrifuged at 14000 g, 4°C for 20 min. The supernatants were spun in a vacuum concentrator until they dry. The dried metabolite pellets were reconstituted by 60% methanol and analyzed by LC-MS/MS, mixing the same amount of supernatant from each processed sample as a QC sample.

*Fecal Collection*. Fecal samples were collected directly from the intestines of each sacrificed rat and placed in sterile EP tubes at the end of week 4 and stored at −80°C.

*HE Staining*. All rats were sacrificed on the 28th day and colon tissues were taken and fixed in neutral paraformaldehyde for 48 hours. 4 *μ*m sections were cut and embedded in paraffin, stained with hematoxylin-eosin, and sealed with neutral gum for observation by light microscope.

### 2.5. Serum UHPLC-MS/MS Analysis

*UHPLC-MS/MS Conditions*. LC-MS/MS analyses were performed using a Vanquish UHPLC system (Thermo Fisher, USA) coupled with an Orbitrap Q Exactive HF-X mass spectrometer (Thermo Fisher, USA) operating in the data-dependent acquisition (DDA) mode. Samples were injected onto an Accucore HILIC column (100 × 2.1 mm, 2.6 *μ*m) using a 16 min linear gradient at a flow rate of 0.3 mL/min. The eluents for the positive polarity mode were eluent A (0.1% FA in 95% ACN, 10 mM ammonium acetate) and eluent B (0.1% FA in 50% ACN, 10 mM ammonium acetate). The eluents for the negative polarity mode were eluent A (95% ACN, 10 mM ammonium acetate, pH 9.0) and eluent B (50% ACN, 10 mM ammonium acetate, pH 9.0). The solvent gradient was set as follows: 2% B, 1.5 min; 2-100% B, 12.0 min; 100% B, 14.0 min; 100-2% B, 14.1 min; 2% B, 16 min. Q Exactive HF-X mass spectrometer was operated in positive/negative polarity mode with spray voltage of 3.2 kV, capillary temperature of 320°C, sheath gas flow rate of 35 arb, and aux gas flow rate of 10 arb.

*Data Processing and Statistical Analysis*. The raw data files generated by UHPLC-MS/MS were processed using the Compound Discoverer 3.0 (CD 3.0, Thermo Fisher, USA) to perform peak alignment, peak picking, and quantitation for each metabolite. After that, peak intensities were normalized to the total spectral intensity. The normalized data was used to predict the molecular formula based on additive ions, molecular ion peaks, and fragment ions. And then peaks were matched with the mzCloud (https://www.mzcloud.org/) and ChemSpider (http://www.chemspider.com/) database to obtain the accurate qualitative and relative quantitative results. PCA and PLS-DA were performed with MetaX software (BGI Tech, China) [17]. Variable Importance Projection (VIP) produced by PLS-DA and Fold Change (FC) were used to screen for differential metabolites with P value of T-test (VIP > 1, FC > 2.0 or FC < 0.5 and P < 0.05). Specificity and sensitivity of identified potential biomarkers were analyzed by ROC curves, and metabolic pathways involving potential biomarkers were topologically analyzed by the MetaboAnalyst 3.0 pathway analysis module (www.metaboanalyst.ca). LC-MS/MS assay was performed by Novogene Co., Ltd. (Beijing, China).

### 2.6. Intestinal Flora Analysis

*Fecal DNA Extraction*. Fecal genomic DNA was extracted using Qiagen QIAamp DNA Stool Mini Kit (Qiagen, Germany). DNA concentration and purity were monitored on 1% agarose gels. According to the concentration, DNA was diluted to 1 ng/*μ*L using sterile water.

*PCR Amplification and Product Purification*. 16S rRNA genes of 16S V4 regions were amplified using specific primer (515F-806R) with the barcode. All PCR reactions were carried out in 30 *μ*L reactions with 15 *μ*L of Phusion® High-Fidelity PCR Master Mix (New England Biolabs, USA), 0.2 *μ*M of forward and reverse primers, and about 10 ng template DNA. Thermal cycling consisted of initial denaturation at 98°C for 1 min, followed by 30 cycles of denaturation at 98°C for 10s, annealing at 50°C for 30s, and elongation at 72°C for 30s and finally 72°C for 5 min. The same volume of 1×loading buffer (contained SYB green) was mixed with PCR products and electrophoresis was operated on 2% agarose gel for detection. PCR products were mixed in equidensity ratios. Then, mixture PCR product was purified with GeneJET™ Gel Extraction Kit (Thermo Scientific, USA).

*Library Preparation and Sequencing Analysis*. Sequencing libraries were generated using Ion Plus Fragment Library Kit 48 rxns (Thermo Scientific, USA) following manufacturer's recommendations. The library quality was assessed on the Qubit@ 2.0 Fluorometer (Thermo Scientific, USA). At last, the library was sequenced on an Ion S5TM XL platform (Thermo Scientific, USA) and 400 bp/600bp single-end reads were generated. The raw reads were spliced and filtered to obtain clean reads, and then all clean reads were clustered by Uparse software (Uparse v7.0.1001), sequences with ≥97% similarity were assigned to the same OTUs, and representative sequence for each OTU was screened for further species annotation through Silva Database (https://www.arb-silva.de/). Alpha diversity was analyzed by Observed Species, Shannon Index, and Chao1. Beta diversity was expressed as PCA. MetaStat and LEfSe methods were used to compare species with significant differences among groups. Spearman correlation coefficient was calculated to figure out the correlation between genus, species, and metabolites. 16S rDNA sequencing was performed by Novogene Co., Ltd. (Beijing, China).

## 3. Results

### 3.1. Blood Pressure and HE Staining

Systolic and diastolic blood pressure in HD group were not significantly different from those in M group before treatment (P > 0.05). After 3 weeks of treatment, the diastolic blood pressure in HD group was significantly lower than that in M group (P < 0.05). After 4 weeks of treatment, both systolic and diastolic blood pressure in HD group were lower than that in M group (P < 0.05) (Figure 1(a)). HE staining showed no significant inflammation and dysplasia in intestinal tissue in three groups (Figure 1(b)). Considering the chronic systemic low-grade inflammatory state in hypertension [3], pathological changes of intestine were not visually identified in HE staining.

### 3.2. Abundance and Diversity of Intestinal Flora

When the sequencing reads approached 80 000, the sequencing reached plateau stage suggesting full sequencing. The number of species was compared with W group > HD group > M group (Figure 2(a)). Chao1 index was proportional to the abundance of intestinal flora and Shannon index was proportional to the diversity of intestinal flora. The abundance and diversity of intestinal flora in M group were all lower than those in W group, both of which recovered with different degrees after administration of HD (Figures 2(b) and 2(c)). Further PCA analysis was conducted based on Euclidean distances (Figure 2(d)), and the data suggested that the aggregation degree of samples in W group and HD group was better than that in M group, indicating that HD improved the disorder of intestinal flora in SHRs.

### 3.3. Screening of Intestinal Differential Flora

We compared the relative abundance of the three groups at the phylum, genus, and species levels. The top 5 phyla among the three groups were Firmicutes, Bacteroidetes, Verrucomicrobia, Actinobacteria, and Tenericutes (Figure 3(a)). In M group, the abundance of Firmicutes increased, the abundance of Bacteroidetes decreased, the ratio of Firmicutes to Bacteroidetes (F/B) increased, and the ratio of F/B recovered after administration of HD (Figures 3(b), 3(c), and 3(d)). We further used LEfSe (LDA score > 3.8) to analyze the statistically significant biomarkers among three groups. The dominant genuses and species of the W group were* Lachnoclostridium, Faecalibaculum, *and* Lactobacillus reuteri*, and the dominant genuses and species were* Akkermansia, Akkermansia muciniphila, *and* Lactobacillus intestinalis *in HD group; however, no dominant genus or species was found in M group (Figure 4(a)). The M group was further compared with the HD group and the W group to find the dominant genus and species. Compared with the HD group, the abundance of* rumen bacterium NK4A214 *was increased, and the abundance of* Akkermansia, Akkermansia muciniphila, *and* Lactobacillus intestinalis* was decreased in M group (Figure 4(b)). Compared with the W group, the abundance of* Clostridium *sp*. MC 40* was increased, and the abundance of* Lachnoclostridium, Faecalibaculum, *and* Lactobacillus reuteri* was decreased in M group (Figure 4(c)).

### 3.4. Metabolic Pattern Recognition and Data Analysis

We analyzed the serum metabolism to validate efficacy of HD. PCA analysis of the total samples showed that the QC samples were clustered, suggesting that the experimental data were well controlled. The metabolic patterns of W group were significantly different from those of HD group and M group (Figures 5(a) and 5(b)). The PCA and PLSDA analysis (Figures 5(c), 5(d), and 5(e)) were further performed in the HD group and the M group, and the metabolic patterns of the two groups were also significantly different. Compared with the M group, R2Y and Q2Y, representing the explanatory and predictive ability of PLSDA model, were close to 1 in W group and HD group, suggesting that the explanatory and predictive value of PLSDA model was high. The data demonstrated there were significant differences between WKY rats and SHRs in serum endogenous metabolites, and the serum metabolism of SHRs also changed significantly after administration of HD.

### 3.5. Identification of Potential Biomarkers

We screened differential metabolites by VIP > 1, FC > 2.0 or FC < 0.5, and P value < 0.05 (Figures 6(a) and 6(b)). Ultimately, 16 potential biomarkers were identified that may be associated with lowering blood pressure (Table 1). Details of the 16 metabolites were presented in the supplementary materials (Table S). Seven metabolites increased and 9 metabolites decreased in M group. 16 metabolites tended to be of normal level after intervention with HD. Receiver operating characteristic (ROC) curves were used to analyze the predictive ability of 16 potential biomarkers. By comparison with M group, all of them demonstrated high prediction accuracy, especially leukotriene B4, testosterone, prostaglandin E2, gamma-aminobutyric acid, arachidonic acid, L-glutathione (reduced), cortisone, and 5-hydroxyindoleacetic acid (Figure 7). Hierarchical clustering analysis of all differential metabolites including 16 potential biomarkers showed that the metabolic patterns and metabolic function of WKY rats and SHRs were different. The metabolic function of serum endogenous metabolites in SHRs changed significantly after the HD intervention (Figures 6(c) and 6(d)). To explore the metabolic function of the 16 potential biomarkers, we ran the pathway analysis module with Metaboanalys software. The results showed that arachidonic acid metabolism, tryptophan metabolism, glutathione metabolism, and steroid hormone biosynthesis were the top 4 enrichment and topological pathways (Table 2, Figure 8).

### 3.6. Correlation between Potential Biomarkers and Differential Flora

Considering intestinal flora can regulate the metabolic function of the host, we compared the correlation of 8 significantly different genuses and species with 16 potential biomarkers using Spearman statistical method.* Akkermansia* and* Akkermansia muciniphila* were highly negatively correlated with indoleacetic acid and testosterone, while* Lactobacillus intestinalis *was highly positively correlated with 5-hydroxyindoleacetic acid and beta-estradiol and highly negatively correlated with indoleacetic acid and prostaglandin E2.* Lachnoclostridium *had a high positive correlation with L-kynurenine and 4-pyridinic acid, and a high negative correlation with arachidonic acid, leukotriene B4, and testosterone, while* Lactobacillus reuteri* was highly negatively correlated with leukotriene B4 and testosterone.* Clostridium *sp.* MC 40 *showed a high negative correlation with L-kynurenine and 4-pyridinic acid, and a high positive correlation with indoleacetic acid, prostaglandin E2, and testosterone (Table 3).

## 4. Discussion

Both our results of the intestinal flora and serum metabolism indicated that HD administration demonstrated protective effects on SHRs. Correlation analysis indicated that the intestinal flora might concentrate on regulating metabolites in certain metabolic pathways, thereby reducing blood pressure.

Firmicutes and Bacteroidetes account for 90% or more in human intestinal flora. The ratio of Firmicutes to Bacteroidetes (F/B) and the richness, diversity, and evenness are important indicators reflecting the disorder of intestinal flora [1–3]. Our results suggested that the dominant phylum in three groups were similar to the human. The richness and diversity decreased and the F/B ratio of SHRs increased compared to those of WKY rats, which was consistent with previous studies in intestinal flora of SHRs and prehypertension and hypertension patients [4, 6]. According to the recovered richness and diversity and decreased F/B ratio after administration of HD, we proposed that HD ameliorated the disorder of the structure and composition in SHRs' intestinal flora to a certain extent.

We further screened for differential flora that might restore intestinal flora disorder and lower blood pressure. The abundance of* Akkermansia*,* Akkermansia muciniphila,* and* Lactobacillus intestinalis* was increased after administration of HD. They were functionally similar to* Lachnoclostridium*,* Faecalibaculum,* and* Lactobacillus reuteri*, which had high abundance in WKY rats.* Lactobacillus intestinalis *has been verified at low level in hyperlipidemic rats and its abundance was inversely correlated with fat content and body weight [18], as well as the increased inflammatory response in rats with spinal cord injury [19].* Lactobacillus reuteri *reduced chronic periodontitis [20] and improved the antioxidant and immune function of piglets [21]. In addition,* Lactobacillus intestinalis* and* Lactobacillus reuteri* all belong to* lactobacillus* producing lactic acid. Wilck et al. reported that high-salt diet decreased the level of* lactobacillus *and increased blood pressure [22]. As a bacteria producing butyric acid,* Akkermansia muciniphila *has been found with less abundance in obese and diabetic mice and patients, which improved hyperlipidemia and insulin resistance, reduced the level of circulating inflammatory factors, reduced endotoxemia, and improved intestinal barrier function [23, 24].* Lachnoclostridium *as a butyrate-producing bacterium also improved obesity and insulin resistance [25, 26].* Faecalibaculum *was a newly isolated genus from mice in recent years and its main metabolic end product was lactic acid [27]. Butyric acid, as the main component of short-chain fatty acids, regulated inflammation and immunity and improved intestinal barrier function [28]. Besides, the increase of butyric acid and lactic acid in the body promoted the abundance of each other's producing bacteria, thus forming a positive feedback loop and increasing the protective effect [29]. Our results identified the notion that the increased* rumen bacterium NK4A214* and* Clostridium *sp.* MC 40* in SHRs belong to* unidentified Ruminococcaceae*, which was not reported before and should be paid attention to. Our results suggested that* Akkermansia*,* Akkermansia muciniphila,* and* Lactobacillus intestinalis* might regulate blood pressure by regulating factors related to elevated blood pressure such as inflammation, blood lipids, and blood sugar. Besides, certain genus and species of Ruminococcaceae might be associated with elevated blood pressure.

Based on the fact that some of the final products of intestinal flora fermentation can enter the blood and exert an important effect on the physiology of the host, we further studied the changes of serum metabolism of SHRs. 16 metabolites were screened out to be related to lowering blood pressure, all of which had very high accuracy of prediction, especially leukotriene B4, testosterone, prostaglandin E2, gamma-aminobutyric acid, arachidonic acid, L-glutathione (reduced), cortisone, and 5-hydroxyindoleacetic acid. We further explored the antihypertensive mechanism through the metabolic pathways involving 16 metabolites, which were mainly enriched in arachidonic acid metabolism, tryptophan metabolism, steroid hormones biosynthesis, and glutathione metabolism.

### 4.1. Arachidonic Acid Metabolism

The content of arachidonic acid (AA), prostaglandin E2 (PGE2), and leukotriene B4 (LTB4) in the arachidonic acid metabolism was all decreased after the administration of HD. AA was a substrate synthesizing a variety of proinflammatory, procoagulant, and vasoconstrictive substances and participating in the pathological process of hypertension [30], which was significantly positively correlated with the prevalence of hypertension and cardiovascular risk [31, 32]. PGE2 binds to its G protein-coupled receptors (GPCR) EP1 and EP3, leading to constricted blood vessels, platelet aggregation, inflammatory reactions, and increased blood pressure [33–35], which was involved in promoting salt-sensitive hypertension [36]. LTB4 is produced by AA via the 5-lipoxygenase (5-LOX)/leukotriene A4 (LTA4)/LTA4 hydrolase (LTA4H) pathway and is widely involved in inflammatory responses [33]. Relevant studies have found that LTB4 injection in SHRs' solitary bundle nucleus (NTS) caused elevated blood pressure, and the blocking of LTB4 receptor 1 (BLT1) significantly decreased blood pressure [37, 38]. HD might achieve the antihypertensive effect through anti-inflammatory, antiplatelet aggregation and vasodilatation by decreasing the level of the three metabolites.

### 4.2. Tryptophan Metabolism

The content of L-kynurenine (L-kyn) and 5-hydroxyindoleacetic acid (5-HIAA) in the tryptophan metabolism increased after administration of HD, while the content of indoleacetic acid (IAA) decreased. Tryptophan is an essential amino acid of the human body, which is decomposed via serotonin (5-HT) and kyn. IAA is a metabolite of the kyn pathway, and 5-HIAA is a metabolite of the 5-HT pathway. Repeated release of 5-HT contracted blood vessels, promoted platelet aggregation, and raised blood pressure [39]. 5-HT serotonin transporter (SERT) could reuptake 5-HT and degrade it into 5-HIAA in intestinal epithelial cells or nerve cells, alleviating the enterotoxicity and neurotoxicity of free 5-HT [40]. Indoleamine 2,3 dioxygenase (IDO) metabolized tryptophan to kyn and thereby decreased the blood pressure of inflammatory mice, while inhibition of IDO activity reduced the generation of kyn and then rebounded blood pressure [41]. Studies has found that kylinase (KYNU) mRNA levels were elevated in SHRs' brainstem, since KYNU catalyzed Kyn as 3-hydroxyanthronic acid (3-HAA), and 3-HAA promoted AA to produce prostaglandin E and leukotriene under the action of Cyclooxygenase 2 (COX2) and 5-LOX, both of which were closely related to the increase of blood pressure [42, 43]. HD might restore the disturbance of L-kyn, 5-HIAA, and IAA by regulating the activities of SERT, IDO, and KYNU in tryptophan metabolism, which probably interact with arachidonic acid in the process of antihypertension.

### 4.3. Steroid Hormone Biosynthesis

Steroid hormones include sex hormones and corticosteroids. After administration of HD, the contents of testosterone and cortisone in SHRs' serum decreased, while the contents of beta-estradiol increased. Testosterone is the main component of androgen and estradiol is the most active component of estrogen. Both testosterone supplementation and reduction of 17 beta-estradiol activated the RAAS system in vivo to increase blood pressure [44, 45]. Cortisone, as a glucocorticoid, promoted the reabsorption of water and sodium in the kidneys and increased blood pressure after being transformed into the active hydrocortisone [46]. Affecting the sex hormones and corticosteroid levels of SHRs may be involved in antihypertensive effect of HD.

### 4.4. Glutathione and Other Metabolism

We also observed that the level of glutathione (reduced), glycine, taurocholic acid, 4-pyridoxic acid, gamma-aminobutyric acid, and sphingosine 1-phosphate increased and adrenic acid decreased after administration of HD. Glycine is one of the components of reduced glutathione, which enhanced the activity of superoxide dismutase (SOD) and glutathione peroxidase (GSH-Px), scavenged oxygen free radicals, and improved the capability against oxidative stress [47, 48]. Taurocholic acid, an important product of bile acid metabolism, reduced liver lipid accumulation [49]. 4-pyridic acid was a metabolite of vitamin B6, and the low level of vitamin B6 was closely related to inflammatory status and cardiovascular mortality [50]. Gamma-aminobutyric acid, as an inhibitory neurotransmitter, has been found to be decreased in salt-sensitive hypertensive rats, and its increase decreased SHRs' blood pressure [51, 52]. Sphingosine 1-phosphate was catalyzed by sphingosine kinase (SPK) through the S1P receptor. The activation of SPK/S1P signaling pathway activated eNOS and protected myocardial cells from acute ischemia-reperfusion [53, 54]. As an omega-6 polyunsaturated fatty acid, adrenic acid acted as an inflammatory mediator as a ligand of immune receptor [55]. These changes of metabolites regulated by HD may participate in the antihypertensive process through anti-inflammatory and antioxidative stress effects.

We further analyzed the correlation between genius, species, and metabolites.* Akkermansia*,* Akkermansia muciniphila*, and* Lactobacillus intestinalis* were highly correlated with testosterone, beta-estradiol, indoleacetic acid, 5-hydroxyindoleacetic acid, and prostaglandin E2, which were enriched in steroid hormone biosynthesis, tryptophan metabolism, and arachidonic acid metabolism. Previous studies have found that excessive androgen exposure during perinatal period reduced the levels of* Akkermansia* and* Lactobacillus* in intestinal and increased blood pressure [56]. Our study also found elevated levels of androgen and decreased estrogen levels in SHRs' serum, and the levels of* Akkermansia*,* Akkermansia muciniphila*, and* Lactobacillus intestines *in SHRs' intestinal decreased, while HD improved the disorder. Testosterone, L-kynurenine, arachidonic acid, leukotriene B4, and 4-pyridinic acid, which were highly associated with the dominant* Lachnoclostridium *and* Lactobacillus reuteri* in WKY rats, were enriched in steroid hormone biosynthesis, arachidonic acid metabolism, tryptophan metabolism, and vitamin B6 metabolism.* Lachnoclostridium* was also highly correlated with vitamin B6 metabolism and tryptophan metabolism in mice with colitis [57], similar to our study in WKY rats. Coincidentally, testosterone, L-kynurenine, indoleacetic acid, prostaglandin E2, and 4-pyridinic acid, which were highly correlated with the dominant* Clostridium *sp.* MC 40 *in SHRs, were also enriched in steroid hormone biosynthesis, tryptophan metabolism, arachidonic acid metabolism, and vitamin B6 metabolism. In our study, the metabolites and their enriched metabolic pathways, which were closely related to the three dominant geniuses and species, were highly concentrated. We therefore speculated that the intestinal flora may be the target of HD administration, thus to regulate steroid hormone biosynthesis, arachidonic acid metabolism, tryptophan metabolism, and vitamin B6 metabolism.

## 5. Conclusion

In conclusion, the present study indicated that the combination of* Astragalus membranaceus* and* Salvia miltiorrhiza* demonstrated good antihypertensive effect, which may be driven by the protective intestinal flora and beneficial metabolites. This study provided new insights into the antihypertensive mechanism of* Astragalus membranaceus* and* Salvia miltiorrhiza*.

## Figures and Tables

**Figure 1:** Blood pressure and HE staining. (a) Systolic and diastolic blood pressure changes in 4-week consecutive administration of HD. Results were compared by one-way ANOVA, *∗* P<0.05 compared with M group. (b) Histological changes of colon tissues in HE staining after 4-week consecutive administration of HD at 400 magnification.

**Figure 2:** Abundance and diversity of intestinal flora. (a) Rarefaction curves of three groups for species number after 80000 random sequences number. The curve in each group was near smooth when the sequencing data were great enough with few new species undetected. ((b) and (c)) Box plot of difference among groups of Chao 1 index (used to assess abundance) and Shannon index (used to assess diversity). P values were from Wilcoxon rank sum test. (d) Principal Component Analysis (PCA) of three groups based on Euclidean distances. The percentage of PC1 and PC2 represented the contribution value of the first and second principal components to the sample difference.

**Figure 3:** Changes of flora at the level of phylum. (a) The top 5 phylum of three groups. ((b) and (c)) Box plot of difference among three groups of Firmicutes and Bacteroidetes. The p value was obtained by the permutation test between groups and the p value was corrected by the Benjamini and Hochberg False Discovery Rate (FDR) method to obtain the q value, *∗∗* q<0.01. (d) The ratio of Firmicutes to Bacteroidetes (F/B) in three groups. Results were compared by one-way ANOVA, *∗* P<0.05.

**Figure 4:** Screening of differential genus and species. A LEfSe analysis along with linear discriminate analysis (LDA) was applied to identify genus and species in three groups. Discriminative biomarkers with an LDA score > 3.8; if one group was missing, it means there were no significant biomarkers in this group. (a) M group vs HD group vs W group (M group missing). (b) M group vs HD group. (c) M group vs W group.

**Figure 5:** Metabolic pattern recognition and data analysis. ((a) and (b)) PCA score plot 3D and 2D of three groups and QC samples. PC1, first principle component score; PC2, second principle component score; PC3, third principle component score. The more aggregated the QC samples were, the higher the quality of experimental data was. Ellipses represented 95% confidence intervals. (c) PCA score plot 3D (group HD vs M). ((d) and (e)) PLS-DA score plot 2D (group HD vs M; group W vs M). R2Y represented the interpretation rate of the second principal component of the model and Q2Y represented the prediction rate of the model.

**Figure 6:** Identification of potential biomarkers. ((a) and (b)) Volcano Plot of differential metabolites (group W vs M; group HD vs M). The size of the dot represented the VIP value and alpha represented the transparency of the dot. Black represented metabolites that were not significantly different, red represented upregulated metabolites, and green represented downregulated metabolites. ((c) and (d)) Hierarchical clustering analysis of differential metabolites (group W vs M; group HD vs M). The clustering of the samples was longitudinal; the clustering of the metabolites was horizontal; the shorter the clustering branches, the more similar the color, and the higher the similarity.

**Figure 7:** Receiver operating characteristic (ROC) curves analysis of potential biomarkers (group W vs M; group HD vs M). The area under the ROC curve was called Area Under Curve (AUC), which was used to assess the sensitivity and specificity of biomarkers for predicting events. We regarded AUC > 0.85 as the bottom line of very high prediction accuracy.

**Figure 8:** Metabolic pathway analysis of potential biomarkers. The color and size of circles were based on P value and pathway impact value, respectively. The larger the circle, the larger the impact factor; the darker the color, the smaller the P value, and the more significant the enrichment.

**Table 1:** 16 potential biomarkers among the three groups.

Identification	Formula	Molecular Weight	RT (min)	Change Trend (HD:M^a^ / W:M^b^)	Pathway
Taurocholic acid	C_26_H_45_NO_7_S	515.2900	14.3	↑ / ↑	Primary bile acid biosynthesis
5-Hydroxyindoleacetic acid	C_10_H_9_NO_3_	191.0580	8.36	↑ / ↑	Tryptophan metabolism
Indoleacetic acid	C_10_H_9_NO_2_	175.0631	9.46	↓ / ↓	Tryptophan metabolism
4-Pyridoxic acid	C_8_H_9_NO_4_	183.0530	5.75	↑ / ↑	Vitamin B6 metabolism
L-Kynurenine	C_10_H_12_N_2_O_3_	208.0748	3.75	↑ / ↑	Tryptophan metabolism
Adrenic acid	C_22_H_36_O_2_	332.2709	15.51	↓ / ↓	Biosynthesis of unsaturated fatty acids
Prostaglandin E2	C_20_H_32_O_5_	352.2247	10.63	↓ / ↓	Arachidonic acid metabolism
Leukotriene B4	C_20_H_32_O_4_	336.2296	12.19	↓ / ↓	Arachidonic acid metabolism
Gamma-Aminobutyric acid	C_4_H_9_NO_2_	103.0632	1.31	↑ / ↑	beta-Alanine metabolism
Testosterone	C_19_H_28_O_2_	288.2088	13.85	↓ / ↓	Steroid hormone biosynthesis
Sphinganine 1-phosphate	C_18_H_40_NO_5_P	381.2641	14.59	↑ / ↑	Sphingolipid metabolism
Arachidonic acid	C_20_H_32_O_2_	304.2399	13.62	↓ / ↓	Arachidonic acid metabolism
Glycine	C_2_H_5_NO_2_	75.0320	6.34	↑ / ↑	Glutathione metabolism
Cortisone	C_21_H_28_O_5_	360.1930	11.22	↓ / ↓	Steroid hormone biosynthesis
Beta-Estradiol	C_18_H_24_O_2_	272.1774	11.83	↑ / ↑	Steroid hormone biosynthesis
L-Glutathione (reduced)	C_10_H_17_N_3_O_6_S	307.0833	1.50	↑ / ↑	Glutathione metabolism

*Note.* ^a^Trends of HD group compared with M group. ^b^Trends of W group compared with M group. ↑: up-regulated. ↓: down-regulated.

**Table 2:** Top 10 metabolic pathways of potential biomarkers.

Pathway name	Total	Hits	p	Log(p)	Holm p	FDR	Impact
Arachidonic acid metabolism	36	3	0.0069239	4.9728	0.56084	0.40424	0.36753
Tryptophan metabolism	41	3	0.0099812	4.6071	0.79849	0.40424	0.10622
Glutathione metabolism	26	2	0.033842	3.3861	1	0.72468	0.36642
Steroid hormone biosynthesis	70	3	0.041817	3.1745	1	0.72468	0.07078
Cyanoamino acid metabolism	6	1	0.066665	2.7081	1	0.72468	0
Biosynthesis of unsaturated fatty acids	42	2	0.080649	2.5176	1	0.72468	0
Taurine and hypotaurine metabolism	8	1	0.087945	2.431	1	0.72468	0
Primary bile acid biosynthesis	46	2	0.094426	2.3599	1	0.72468	0.05952
Methane metabolism	9	1	0.098413	2.3186	1	0.72468	0
Vitamin B6 metabolism	9	1	0.098413	2.3186	1	0.72468	0

*Note. *Total: the number of all metabolites in this pathway; Hits: The number of differential metabolites hitting this pathway; Raw p: P value obtained by enrichment analysis; Holm P: P value corrected by Holm-Bonferroni method; Impact: Impact factor from topological analysis.

**Table 3:** Correlation between potential biomarkers and differential flora (Rho value / P value).

	*Akkermansia*	*Lactobacillus intestinalis*	*Akkermansia muciniphila*	*Rumen bacterium NK4A214*	*Lachnoclostridium*	*Faecalibaculum*	*Lactobacillus reuteri*	*Clostridium sp. MC 40*
Taurocholic acid	0.605/0.013	0.653/0.0	0.607/0.013	-0.385/0.141	0.094/0.729	0.462/0.072	0.556/0.025	-0.441/0.088
L-Kynurenine	0.330/0.212	0.515/0.017	0.314/0.008	-0.579/0.154	0.753/0.001*∗*	0.691/0.003	0.582/0.018	-0.758/0/0007*∗*
5-Hydroxyindoleacetic acid	0.639/0.008	0.709/0.002*∗*	0.651/0.006	-0.391/0.134	0.432/0.094	0.224/0.405	0.218/0.418	-0,276/0.3
Indoleacetic acid	-0.728/0.001*∗*	-0.829/0.00007*∗*	-0.729/0.001*∗*	0.55/0.027	-0.679/0.004	-0.671/0.004	-0.559/0.024	0.73/0.001*∗*
4-Pyridoxic acid	0.265/0.321	0.459/0.074	0.242/0.367	-0.482/0.058	0.715/0.002*∗*	0.662/0.005	0.568/0.0022	-0.729/0.001*∗*
Adrenic acid	-0.509/0.044	-0.638/0.008	-0.520/0.039	0.588/0.017	-0.662/0.005	-0.482/0.058	-0.524/0.037	0.56/0.024
Arachidonic acid	-0.437/0.090	-0.388/0.137	-0.436/0.091	0.368/0.161	-0.75/0.001*∗*	-0.518/0.040	-0.594/0.015	0.699/0.003
Prostaglandin E2	-0.631/0.009	-0.709/0.002*∗*	-0.617/0.011	0.4/0.125	-0.641/0.007	-0.641/0.007	-0.685/0.003	0.736/0.001*∗*
Leukotriene B4	-0.681/0.004	-0.676/0.004	-0.679/0.004	0.359/0.172	-0.741/0.001*∗*	-0.635/0.008	-0.774/0.0004*∗*	0.677/0.004
Gamma-Aminobutyric acid	0.453/0.078	0.415/0.110	0.476/0.063	-0.379/0.147	0.579/0.019	0.403/0.122	0.344/0.192	-0.504/0.046
Sphinganine 1-phosphate	0.260/0.330	0.674/0.004	0.264/0.324	-0.3/0.259	0.624/0.010	0.485/0.057	0.568/0.022	-0.582/0.018
Glycine	0.471/0.066	0.435/0.092	0.474/0.063	-0.282/0.289	0.518/0.040	0.241/0.368	0.321/0.226	-0.415/0.11
Cortisone	-0.472/0.065	-0.547/0.028	-0.467/0.068	0.485/0.057	-0.45/0.080	-0.25/0.350	-0.35/0.184	0.554/0.026
Testosterone	-0.726/0.001*∗*	-0.471/0.066	-0.726/0.001*∗*	0.35/0.184	-0.721/0.002*∗*	-0.697/0.003	-0.715/0.002*∗*	0.782/0.0003*∗*
Beta-Estradiol	0.506/0.045	0.738/0.001*∗*	0.508/0.044	-0.3/0.259	0.438/0.090	0.362/0.169	0.497/0.05	-0.424/0.101
L-Glutathione (reduced)	0.677/0.004	0.656/0.006	0.677/0.004	-0.415/0.110	0.426/0.099	0.218/0.418	0.215/0.425	-0.285/0.284

*Note ∗* indicates |rho|≥0.7, p<0.05, which is considered to be highly correlated and statistically significant.

## Data Availability

The data used to support the findings of this study are included within the article. If additional support data are needed, they are available from the corresponding author or first author upon request. First author's mailbox is hancong_kidney@hotmail.com. Corresponding author's mailbox is lweidw@163.com.

## Supplementary Materials

Supplementary Materials Details of the 16 metabolites were presented in the supplementary materials (Table S).
